# Associations between *PHACTR1* gene polymorphisms and pulse pressure in Chinese Han population

**DOI:** 10.1042/BSR20193779

**Published:** 2020-06-05

**Authors:** Kunfang Gu, Yue Zhang, Ke Sun, Xiubo Jiang

**Affiliations:** Department of Epidemiology and Health Statistics, the School of Public Health of Qingdao University, No. 38 Dengzhou Road, Qingdao 266021, China

**Keywords:** haplotype, interaction, PHACTR1, polymorphism, pulse pressure

## Abstract

A genome-wide association study (GWAS) in Chinese twins was performed to explore associations between genes and pulse pressure (PP) in 2012, and detected a suggestive association in the phosphatase and actin regulator 1 (*PHACTR1*) gene on chromosome 6p24.1 (rs1223397, *P*=1.04e^−07^). The purpose of the present study was to investigate associations of *PHACTR1* gene polymorphisms with PP in a Chinese population. We recruited 347 subjects with PP ≥ 65 mmHg as cases and 359 subjects with 30 ≤ PP ≤ 45 mmHg as controls. Seven single nucleotide polymorphisms (SNPs) in the *PHACTR1* gene were genotyped. Logistic regression was performed to explore associations between SNPs and PP in codominant, additive, dominant, recessive and overdominant models. The Pearson’s χ^2^ test was applied to assess the relationships of haplotypes and PP. The A allele of rs9349379 had a positive effect on high PP. Multivariate logistic regression analysis showed that rs9349379 was significantly related to high PP in codominant [AA vs GG, 2.255 (1.132–4.492)], additive [GG vs GA vs AA, 1.368 (1.049–1.783)] and recessive [AA vs GA + GG, 2.062 (1.051–4.045)] models. The positive association between rs499818 and high PP was significant in codominant [AA vs GG, 3.483 (1.044–11.613)] and recessive [AA vs GG + GA, 3.716 (1.119–12.339)] models. No significant association of haplotypes with PP was detected. There was no significant interaction between six SNPs without strong linkage. In conclusion, the present study presents that rs9349379 and rs499818 in the *PHACTR1* gene were significantly associated with PP in Chinese population. Future research should be conducted to confirm them.

## Introduction

Pulse pressure (PP) is the difference between systolic blood pressure (SBP) and diastolic blood pressure (DBP), reflecting the fluctuation of blood pressure during each cardiac contraction [1,2]. Widening PP is an independent risk factor for coronary heart disease (CHD), myocardial infarction (MI), stroke and is linked to mortality [3–6]. Studies have demonstrated that some environmental factors affect PP. For instance, reduced arterial compliance in large arteries with age leads to elevated PP [7]. Gender affects PP through changing the time for return of the reflected wave, dependent on body height [8]. In addition, PP might be influenced by cholesterol, diabetes and hypertension [2].

Besides the above environmental factors, PP is related to genetic factors. Genetic epidemiological studies using families or twins have reported a series of data on the heritability estimates of PP, ranging from 0.11 [9] in black African families to 0.63 [10] in Swedish families [9–25]. Among them, a study of Chinese twins displayed that the heritability estimate is 0.45 [11], which is similar to Polish (0.37) [12] and American (0.51) [21] studies using family data, respectively.

Recent studies have increasingly demonstrated that phosphatase and actin regulator 1 (*PHACTR1*) gene polymorphisms are associated with cardiovascular disease (CVD) in different populations, including Mexicans, Caucasians and Chinese, etc. [26–37]. Of note, a genome-wide linkage and genome-wide association study (GWAS) for PP in Chinese twins was performed in 2012. The present study identified a suggestive linkage peak on chromosome 6 (LOD score = 3.19) and found a suggestive association between rs1223397 in chromosome 6p24.1 *PHACTR1* gene and PP (*P*=1.04e^−07^) [5].

The product of the *PHACTR1* gene is a binding protein of protein phosphatase 1 (PP1) and actin via four RPEL-repeat sequences [38,39]. As a regulator of PP1 activity, PHACTR1 is highly expressed in endothelial cells (ECs) of the brain and heart, playing an important role in regulating endothelial tubulogenesis, motility and apoptosis [34,39–41]. It is also expressed in ECs of arteries and is related to altered vasomotor properties [32,37,42]. Considering the regulating function of PHACTR1 and the independent contribution of PP to cardiovascular and cerebrovascular diseases, we wondered whether polymorphisms of the *PHACTR1* gene contribute to the susceptibility of high PP.

Therefore, we performed the present study to examine the associations between *PHACTR1* gene polymorphisms and PP in a Chinese population.

## Materials and methods

### Study participants

The case–control study was performed from July 2015 to December 2017, among subjects residing in four districts (Shibei, Shi’nan, Huangdao, Licang) of Qingdao, China. Participants aged 30 years and over and trained investigators completed the questionnaires on a face to face basis. All participants recruited were ethnic Han permanent residents. Patients with an antecedent or current history of cancer, valvular diseases, cardiovascular and cerebrovascular diseases (CHD, MI and stroke, etc), and severe hepatorenal disease were excluded. In addition, pregnant or lactating women were excluded. The case group consisted of subjects with PP ≥ 65 mmHg. The control group included individuals with 30 ≤ PP ≤ 45 mmHg, SBP ≤ 120 mmHg and DBP ≤ 80 mmHg, excluding those with antihypertensive medication currently. A total of 706 blood samples (347 cases and 359 controls) were successfully collected and genotyped.

The research complied with the Declaration of Helsinki and was supported by the Ethics Committee of Qingdao University Medical College. Every participant provided written informed consent.

### Single nucleotide polymorphisms selection and genotyping

The selection of single nucleotide polymorphisms (SNPs) was based on the Chinese Han Beijing (CHB) population data of HapMap (HapMap Data Rel 27 PhaseII + III) and 1000 Genomes Project database (http://browser.1000genomes.org/index.html). We used Haploview 4.2 software (https://www.broadinstitute.org/haploview/downloads) to screen tag-SNPs according to minor allele frequency (MAF) > 0.05 and r^2^ > 0.8. In addition, we screened the literature of SNPs related to blood pressure or CVD in PubMed and Google [5,26–29,31,34,43–45]. Finally, seven SNPs in the *PHACTR1* gene were selected for the present study, i.e., rs475543, rs9472419, rs2026458, rs9349379, rs1223397, rs693758, rs499818.

Genomic DNA was extracted from the peripheral blood of each subject using DNA isolation kits (BioTeKe Corpration, Beijing) and stored at −20°C before genotyping. SNPs genotyping was provided by the Bio Miao Biological Technology (Beijing) Co., Ltd using Matrix-Assisted Laser Desorption/Ionization Time of Flight Mass Spectrometry (MALDI TOF–MS) of the MassARRAY system (Sequenom Inc., San Diego, CA, U.S.A.). The design of PCR primers was performed by Assay Design 3.1 software (Sequenom Inc., San Diego, CA, U.S.A.) and listed in Supplementary File S1. Genotyping was carried out without knowing the case or control status of blood samples for quality control. We randomly selected 10% of samples for repeated genotyping detection, and the consistency of the results was more than 99%.

### Definitions

In the present study, we adopted body mass index (BMI) proposed by China to diagnose obesity (non-obese < 28 kg/m^2^; obese ≥ 28 kg/m^2^) [46]. According to the Chinese adult dyslipidemia prevention guide (2016), dyslipidemia was defined as meeting one of the following criteria: (i) total cholesterol (TC) ≥ 5.2 mmol/l; (ii) triglyceride (TG) ≥ 1.7 mmol/l; (iii) high-density lipoprotein cholesterol (HDL-C) < 1.0 mmol/l; (iv) low-density lipoprotein cholesterol (LDL-C) ≥ 3.4 mmol/l [47]. LDL-C level was calculated by the Friedewald equation: LDL-C (mmol/l) = TC–HDL-C–(TG/2.2) (mmol/l) [48]. Diabetes, defined as fasting plasma glucose (FPG) was ≥ 7.0 mmol/l, or 2-h plasma glucose (2h PG) was ≥ 11.1 mmol/l or self-reported physician diagnosis of diabetes history [49]. Smoked ≥ 100 cigarettes in life and currently smoking was defined as smoking, smoked < 100 cigarettes in life or no smoking for 2 years or more was defined as no smoking. Drinking alcohol within the last 6 months was considered alcohol consumption [50]. Recreational activity refered to running, playing ball, swimming, dancing etc.

### Statistical analysis

In the current study, Stata 15.0 (Stata Corp LLC, College Station, TX, U.S.A.) was used for statistical processing of data. The Student’s *t* test was performed to investigate the difference in continuous variables of normal distribution between the cases and controls; if not, the Wilcoxon rank sum test was applied. The formula of Student’s *t* test was as follows:

$$\text{t}=\frac{{\bar{X}}_{1}-{\bar{X}}_{2}}{\sqrt{\frac{(n_{1}-1)S_{1}^{2}+(n_{2}-1)S_{2}^{2}}{n_{1}+n_{2}-2}\left(\frac{1}{n_{1}}+\frac{1}{n_{2}}\right)}}$$

S_1_^2^ and S_2_^2^ were the variance of two samples, n_1_ and n_2_ were the number of two samples.

Pearson’s χ^2^ test was used to compare the difference of categorized variables between groups and verify the Hardy–Weinberg Equilibrium (HWE). The formula of Pearson’s χ^2^ test was as follows:

$$\chi^{2}=\sum \frac{{\left(A-T\right)}^{2}}{T}$$

A is the actual frequency; T is the theoretical frequency.

Five genetic models (i.e. codominant, additive, dominant, recessive and overdominant models) were adopted for analysis. To examine the associations between SNPs in the *PHACTR1* gene and PP in five genetic models, odds ratios (ORs) with 95% confidence intervals (CIs) were computed by univariate and multivariate logistic regression. The formula of logistic regression analysis was as follows:

$$\log\text{it}p=\text{In}\left(\frac{p}{1-p}\right)=\beta_{0}+\beta_{1}X_{1}+\beta_{2}X_{2}+\cdots +\beta_{k}X_{k}$$

Based on the univariate analysis, the variables with statistically significant distribution differences between groups were selected as covariates for adjustment in the multivariate logistic regression analysis (including age, BMI, dyslipidemia, diabetes, drinking status and recreational activity). In addition, according to previous literature studies, the multivariate logistic regression analysis also adjusted for gender. The Akaike information criterion (AIC) was applied to determine the optimal inheritance model for each SNP.

Haploview 4.2 software was utilized to conduct pairwise linkage disequilibrium (LD) analysis, construct haplotype blocks and calculate haplotype frequencies. D′ value was greater than 0.75, indicating the presence of strong LD among the SNPs. Haplotypes with total frequency less than 5% were omitted. Pearson’s χ^2^ test was used to compare the distribution of haplotype frequencies between groups. Generalized multifactor dimensionality reduction (GMDR) 0.9 software (http://www.ssg.uab.edu/gmdr/) was used for gene–gene interaction analysis. If there was a strong LD between several SNPs, the SNP with maximum MAF was included in the GMDR model. To control the influence of confounding factors on the results, age, gender, BMI, dyslipidemia, diabetes, drinking status and recreational activity were adjusted as covariates. The cross-validation consistency (CVC), testing balanced accuracy and sign test were applied to evaluate each selected interaction. The CVC score, as a measure of the degree of consistency, was used to determine the best model. The testing balanced accuracy was used to measure the degree to which the interaction accurately predicts case-control status with a score ranging from 0.5 to 1.0. The sign test for prediction accuracy was applied to determine whether the identified model was significant or not. All probabilities (*P*-values) mentioned above were two-sided with *P* less than 0.05 were considered significant.

### Sample power calculation

Quanto 1.2.4. software (http://biostats.usc.edu/software) was used for power analysis based on the following parameter setting: OR was 1.5, the prevalence of high PP was 15% [51–53], type I error rate (α) was 0.05, inheritance model was additive model, and sample size was 706 including 347 cases and 359 controls. Depending on the MAF in the study (range: from 0.09 to 0.48), the power of the study was 62.3–96.3%. The power of the study had reached more than 80% when MAF was 0.15.

## Results

### Demographic characteristics analysis

In the present study, a total of 706 subjects including 347 high PP subjects (cases) and 359 normal PP subjects (controls) were selected. The demographic characteristics of case and control groups are presented in Table 1. Compared with the controls, the high PP group had significant higher age (*P*=0.002). Except for gender and smoking status, there were significant differences in the distribution of BMI, dyslipidemia, diabetes, drinking status and recreational activity between the case and control groups.

**Table 1:** The characteristics of study subjects

Variables	High PP group (*n*=347)	Normal PP group (*n*=359)	*P*-value
Age (years)	54.990 ± 8.138	53.090 ± 8.231	0.002^1^
Gender (Male/Female)	123 (35.4)/224 (64.6)	133 (37.0)/226 (63.0)	0.658^2^
BMI (<28/≥28 kg/m^2^)	244 (70.3)/103 (29.7)	330 (91.9)/29 (8.1)	<0.001^2^
Dyslipidemia (No/Yes)	109 (31.4)/238 (68.6)	159 (44.3)/200 (55.7)	<0.001^2^
Diabetes (No/Yes)	258 (74.6)/88 (25.4)	340 (94.7)/19 (5.3)	<0.001^2^
Smoking status (No/Yes)	292 (84.1)/55 (15.9)	311 (86.6)/48 (13.4)	0.351^2^
Drinking status (No/Yes)	277 (79.8)/70 (20.2)	315 (87.7)/44 (12.3)	0.004^2^
Recreational activity (No/Yes)	336 (96.8)/11 (3.2)	320 (89.1)/39 (10.9)	<0.001^2^

Data are expressed as mean ± standard deviation mean (SD) or frequency (percentage).

1 Student’s *t* test.

2 Pearson’s χ^2^ test.

### Single SNP analysis of *PHACTR1* gene and PP

Details for every SNP in our study are shown in Table 2. Genotype frequencies for all SNPs conformed to HWE in the control samples. The association between each allele and PP, the associations of SNPs with PP in codominant, additive, dominant, recessive and overdominant models are listed in Supplementary File S2. The A allele of rs9349379 had a positive effect on high PP [A vs G, 1.293 (1.016–1.646)]. The univariate logistic regression presented that rs9349379 was correlated with an increased risk of high PP in codominant [AA vs GG, 2.137 (1.129–4.044)], additive [GG vs GA vs AA, 1.290 (1.014–1.641)] and recessive [AA vs GA + GG, 2.029 (1.085–3.793)] models. Besides, the positive association between rs499818 and high PP was significant in codominant [AA vs GG, 3.250 (1.046–10.099)] and recessive [AA vs GG + GA, 3.454 (1.115–10.670)] models.

**Table 2:** SNPs of the *PHACTR1* gene investigated in the present study

SNP ID	Chr	Chr position (GRCh38.p12)	Location	Alleles (major/minor)	MAF (case/control)	HWE *P*^1^
rs475543	6	12717924	Intron 1	G/A	0.11/0.11	0.889
rs9472419	6	12718269	Intron 1	C/T	0.32/0.35	0.449
rs2026458	6	12825642	Intron 3	T/C	0.48/0.46	0.712
rs9349379	6	12903725	Intron 3	G/A	0.28/0.23	0.852
rs1223397	6	13270713	Intron 10	G/C	0.22/0.21	0.618
rs693758	6	13287168	3′UTR	G/A	0.09/0.09	1.000
rs499818	6	13332235	3′near	G/A	0.15/0.14	0.482

1 The HWE *P*-value shows the HWE test in control subjects.

In the multivariate logistic regression analysis, adjusted for age, gender, BMI, dyslipidemia, diabetes, drinking status and recreational activity, the association of rs9349379 in the above three genetic models with the higher possibility of high PP did not change significantly. The adjusted OR (95% CI) for rs9349379 in codominant, additive and recessive models were 2.255 (1.132–4.492), 1.368 (1.049–1.783) and 2.062 (1.051–4.045), respectively. Similarly, there was not signifcant change in the association between rs499818 and PP in codominant [AA vs GG, 3.483 (1.044–11.613)] and recessive [AA vs GG + GA, 3.716 (1.119–12.339)] models.

According to the AIC, corresponding best model for rs9349379 and rs499818 was the codominant model. No significant association between other *PHACTR1* SNPs and PP was found in the present study.

### Haplotype analysis of *PHACTR1* gene

As shown in Figure 1, LD analysis between seven SNPs in the *PHACTR1* gene presented that there was a strong LD between rs475543 and rs9472419, which constructed a haplotype block. The results of haplotype analysis displayed that no significant association of haplotypes with PP was observed (Table 3).

**Figure 1:** The haplotype structure of seven *PHACTR1* SNPs in the total 706 ethnic Han Chinese subjects A haplotype block was determined through the Haploview program. The rs number (top; from left to right) corresponds to the SNP ID and the level of pairwise. Numbers in the squares refer to pairwise LD represented as 100 × D′ values.

**Table 3:** Association of the *PHACTR1* haplotypes and PP

Haplotype^1^	rs475543	rs9472419	Freq (total)	Freq (case)	Freq (control)	**χ**^2^	*P*^2^	Permutation^3^
H1	G	C	0.557	0.568	0.547	0.594	0.441	0.738
H2	G	T	0.334	0.321	0.347	1.029	0.310	0.609
H3	A	C	0.108	0.111	0.106	0.095	0.758	0.952

1 Haplotypes with total frequency less than 5% were omitted.

2 *P*-value for the χ^2^ test.

3 *P*-value for the 1000 permutation test.

### Gene–gene interaction analysis

The GMDR method, adjusted for the above-mentioned covariates, was applied to analyze the interaction among the six SNPs without strong linkage (rs9472419, rs2026458, rs9349379, rs1223397, rs693758, rs499818) in the *PHACTR1* gene. The best interaction combination was a five-locus model with a maximum CVC (10/10), testing accuracy of 48.51% and *P*-value of 0.8281 (Table 4). The result suggested that there was no significant interaction between six SNPs in the study of PP.

**Table 4:** Best gene–gene interaction models, as identified by GMDR

Locus no.	Best combination^1^	Testing accuracy	CVC	*P*
2	rs2026458 rs9349379	0.5011	7/10	0.3770
3	rs9472419 rs2026458 rs9349379	0.4823	6/10	0.6230
4	rs9472419 rs2026458 rs9349379 rs499818	0.4920	7/10	0.8281
5	rs9472419 rs2026458 rs9349379 rs1223397 rs499818	0.4851	10/10	0.8281
6	rs9472419 rs2026458 rs9349379 rs1223397 rs 693758 rs499818	0.4613	10/10	0.8281

1 Adjusting for age, gender, BMI, dyslipidemia, diabetes, drinking status, recreational activity.

## Discussion

The complex etiology of elevated PP is intimately involved with environmental and multigenic factors. Previous studies have revealed that PP is closely associated with polymorphisms of many genes, such as endothelial nitric oxide synthase (*eNOS*) gene, angiotensin-converting enzyme (*ACE*) gene and fibrillin-1 gene [54–57]. With regard to the *PHACTR1* gene, studies have found that rs9369640 was related to hypertension [45], rs1223397 was suggestively associated with PP [5], and rs9349379 was linked to SBP [58]. In this study, we explored the associations of seven SNPs in the *PHACTR1* gene and PP in a Chinese population. The findings displayed that the A allele of rs9349379 was a risk factor for high PP, AA genotype of rs9349379 (located in intron 3) and AA genotype of rs499818 (located in 3′ near) were significantly related to increased possibility of high PP in the best genetic models.

The *PHACTR1* gene is composed of 20 exons and 19 introns, encoding PHACTR1, a 484-amino acid long regulatory protein and member of the phosphatase and actin regulatory proteins family [37,39,59,60]. More studies have displayed that the polymorphisms of the *PHACTR1* gene have been related to the pathogenesis of endothelial dysfunction and vascular diseases, i.e., CHD, MI and hypertension, etc. [26,32,45,61], and endothelial dysfunction makes an important contribution to high PP [62]. Therefore, the association of *PHACTR1* gene polymorphisms with PP may be explained by its influence on the physiological function of vascular EC.

PHACTR1 is thought to be an effective inhibitor of PP1 – a multifunctional enzyme that regulates various cellular processes through dephosphorylating serine and threonine residues of different substrates [41]. Reduced PP1 restricts the dephosphorylation of eNOS to impair the synthesis of nitric oxide (NO) in EC [37,63], which is crucial for normal endothelial function and vascular homeostasis, including modulation of vasomotion and local cell growth [64]. Additionally, Rodríguez-Pérez et al*.* found that intronic polymorphisms in the *PHACTR1* gene might cause abnormal PHACTR1 protein through selective splicing in EC, which predisposes individuals to endothelial dysfunction [65].

Studies on rs9349379 of the *PHACTR1* gene have provided vital evidence for the relationship between the *PHACTR1* gene polymorphisms and the function of EC. Surendran et al*.* thought that the G allele of rs9349379 was linked to lower SBP [58]. It may be due to the G allele of rs9349379 up-regulates the expression of endothelin-1 (*EDN1*) gene, located 600 kb upstream of the *PHACTR1* gene [61]. Increased protein product (ET-1) of the *EDN1* gene combines with endothelin B (ETB) receptors on ECs in great vessels, resulting in endothelium-dependent vasodilation via NO synthesis [66,67]. This may be why individuals with the A allele of rs9349379 had a higher probability of high PP than those with the G allele of rs9349379 in our study. ET-1 could also lower blood pressure through enhancing the excretion of Na and water via ETB receptors in renal collecting system [61,68].

On the other hand, rs9349379 is located at a predicted binding site for the transcriptional activator myocyte enhancer factor-2 (MEF2) [69]. MEF2 is expressed in developing EC and is essential for EC proliferation, survival and vascular endothelial integrity [69,70]. In research by Beaudoin et al., the authors observed that the G allele of rs9349379 disrupted the MEF2-binding motif, reducing PHACTR1 expression levels on EC in the right coronary arteries [71]. In this study, rs9349379 genetic association result is consistent with the above physiology, maybe it is also a possible way to explain the effect of rs9349379 on PP.

Regarding rs499818, previous studies reported that it was linked to MI, stroke, fatal ischemic heart disease and sudden cardiac death [26,72,73], but did not mention the possible mechanism about rs499818. In the present study, there was a significant relationship between genotype of rs499818 and PP in codominant and recessive models, but the difference in allele distribution was not significant between the case and control groups. Duplication studies are needed to confirm the real correlation between SNP and PP.

There are some limitations in our study that should be considered. First, this research was a community-based case–control study. There might be recalls bias and it might affect the results. Second, since the etiology of high PP is complex, other unobserved variables may influence the outcome. Finally, the applicability of the results in the present study to other races needs further validation.

In summary, the present study shows that two SNPs in the *PHACTR1* gene (rs9349379, rs499818) may influence the susceptibility to high PP in a Chinese Han population. Our results provide a new direction for genetic research and mechanism exploration on PP. Large sample size and multiethnic studies should be conducted to confirm the findings.

## Abbreviations

AIC: Akaike information criterion
BMI: body mass index
CHD: coronary heart disease
CI: confidence interval
CVC: cross-validation consistency
CVD: cardiovascular disease
DBP: diastolic blood pressure
EC: endothelial cell
EDN1: endothelin-1
eNOS: endothelial nitric oxide synthase
ETB: endothelin B
GMDR: generalized multifactor dimensionality reduction
GWAS: genome-wide association study
HDL-C: high-density lipoprotein cholesterol
HWE: Hardy–Weinberg Equilibrium
LD: linkage disequilibrium
LDL-C: low-density lipoprotein cholesterol
MAF: minor allele frequency
MEF2: myocyte enhancer factor-2
MI: myocardial infarction
NO: nitric oxide
OR: odds ratio
*PHACTR1*: phosphatase and actin regulator 1
PP: pulse pressure
PP1: protein phosphatase 1
SBP: systolic blood pressure
SNP: single nucleotide polymorphism
TC: total cholesterol
TG: triglyceride
